RETRACTED

# Association between Mutation in SMARCAD1 and Basan Syndrome with Cutaneous Squamous Cell Carcinoma

**DOI:** 10.1155/2022/7840710

**Published:** 2022-05-10

**Authors:** Ying Xiong, Ting Chen, Jia Yu, He Zhou, Baozhen Lu, Lijie Chen, Liwei Sun, Can Wang, Sujun Li, Bo Wu

**Affiliations:** ^1^Department of Dermatology, Affiliated Shenzhen Maternity & Child Healthcare Hospital, Southern Medical University, Shenzhen, Guangdong, China; ^2^Shenzhen Mass Medical Co., Ltd., Shenzhen, Guangdong, China; ^3^Shenzhen Dengding Biopharma Co., Ltd., Shenzhen, Guangdong, China; ^4^Translational Medicine Institute of Jiangxi, The First Affiliated Hospital of Nanchang University, Nanchang, Jiangxi, China

## Abstract

**Background:**

Basan syndrome is a rare autosomal-dominant ectodermal dysplasia with certain clinic-pathological features caused by mutations in the SMARCAD1 gene. Currently, no skin malignancy related to Basan syndrome has been reported. This study was aimed at identifying related gene mutations in a new Chinese pedigree with Basan syndrome and discovering the possible association between Basan syndrome and cutaneous squamous cell carcinoma (cSCC).

**Methods:**

We report a case of Basan syndrome from China with family history of cSCC. The pedigree contains 28 individuals. Among them, 12 members had Basan syndrome, while 4 affected members were diagnosed with cSCC in the 1st and 2nd generations. Whole exome sequencing (WES) and Sanger sequencing were performed for 7 available individuals. The specific gene mutation on pre-mRNA splicing was also analyzed using *in vitro* Minigene assay. In addition, sequencing data was analyzed with bioinformatics workflow, aiming to discover the gene associated with cSCC.

**Results:**

Gene sequencing results showed a heterozygous mutation, c.378+5G>A, in the SMARCAD1 gene in all tested individuals with Basan syndrome. Minigene result implicated the specific mutation may cause splicing variations by exon skipping occurring in the targeted exons.

**Conclusion:**

To the best of our knowledge, this is the first study reported Basan syndrome with family history of cSCC. Despite in this study we cannot draw any conclusion about the association between Basan syndrome and cSCC at the genetic level, this study encourages future works to substantiate this potential but important issue.

## 1. Introduction

Basan syndrome is a rare autosomal-dominant ectodermal dysplasia. After the individual is born, the major clinical manifestations of this disease include facial multiple eruptive milia, palmoplantar blisters and keratoderma, no sweat or fingerprint in the palmoplantar region, and onychodystrophy. The first pedigree with Basan syndrome, an Irish American family, was reported by Dr. Baird in 1964 [1]. As at 2021, only about 14 cases had been documented in literature [1–12].

RETRACTED

Basan syndrome is caused by a mutation in the SMARCAD1 gene. By using the first-generation sequencing, Marks et al. detected a heterozygous mutation in the SMARCAD1 gene: c.378+3A>T. They believed this gene is likely to be the pathogenic gene of Basan syndrome [5]. In 2016, Dr. Li's team in China discovered a new gene site, c.378+1G>T, in a Chinese family with Basan syndrome using whole genome sequencing [6]. In 2017 and 2018, Chang et al. and Valentin et al. discovered mutations at new gene sites: c.378+5G>A and c.378+2T>G [2, 7]. It is worth noting that all 4 mutations mentioned above are at the same conservative splicing site in the SMARCAD1 gene. It is difficult to demonstrate any difference of those segregated mutations by simulating the real-world situation in vitro [5, 13]. However, less is known about the mechanism of splice site mutations of SMARCAD1 gene.

Now, we are reporting a new Chinese pedigree with Basan syndrome and family history of cutaneous squamous cell carcinoma (cSCC). To the best of our knowledge, no previous study has found the correlation between Basan syndrome and malignant cutaneous tumors. We aimed to identify pathogenic gene mutations in Basan syndrome and try to discover the possible association between Basan syndrome and cSCC.

## 2. Methods

The study was approved by the IRB of the Affiliated Shenzhen Maternity & Child Healthcare Hospital, Southern Medical University with case ID “Shenzhen Maternity & Child Healthcare Hospital Academic Review (2021) No. 43.” Written consent forms were acquired from all participated family members.

### 2.1. Proband

The proband is a female aged 1 year and 4 months. At the time the proband was born, she exhibited facial multiple eruptive milia, mostly concentrating on the chin (Figure 1(a)). One week later, small (rice-sized) scattered blisters appeared at the end of hands and feet. The majority of blisters were in the palmoplantar region. A few small blisters also fused into larger ones. Later, blisters on hands and feet gradually ruptured and healed, while mild hyperpigmentation and skin atrophy gradually emerged. The proband exhibited no sweat or fingerprint on hands and feet. At the same time, hyperkeratosis, skin atrophy, and mild pigmentation in the palmar-plantar region can be observed (Figure 1(b)).

### 2.2. Pedigree Investigation

Several family members of the proband had the similar rash, including the father, grandfather, and great-grandfather.  Figure 1 shows lack of fingerprint (Figure 1(c)), longitudinal ridges of nails (Figure 1(d)), and obvious hyperkeratosis in the plantar region of the proband's father (Figure 1(e)).

RETRACTED

We investigated 4 generations in the proband's family. With the approval of the Institutional Review Board and consents of the proband's parents and other family members, we obtained 7 individuals' blood samples for genetic tests, including the proband, the parents, and 4 other family members (Figure 2, III-2, III-6, III-10, III-11, IV-1, IV-4, and IV-6).

### 2.3. Whole Exome Sequencing (WES) and Sanger Sequencing

Several previous studies have revealed the pathogenic gene of Basan syndrome: the SMARCAD1 gene [2, 5–7]. Therefore, in this study, we also targeted on this gene. We used the Berry Custom Design V2 to capture and enrich the target gene exons and adjacent splicing regions. We performed the sequencing on the NovaSeq 6000 platform. The raw data yielded 15.75 GB. The average depth of the target region was 117.77×. We designed specific primers for the exons where a mutation at the candidate pathogenic gene site is located. We also performed Sanger sequencing for the target gene. Chromas software was employed to analyze sequencing peaks.

### 2.4. Sequencing Analysis Workflow

We used the Trimmomatic software to filter the raw data. Then, we used the GRCh38 genome as the reference genome. BWA was employed to map the clean reads. The GATK was used for variant discovery. We performed the germline variant calling and variant filtering by germline short variant discovery in the GATK package. Finally, Founctator was employed for variants annotations.

### 2.5. Minigene

#### 2.5.1. Plasmid Construction

*In vitro* Minigene splicing assay was carried out to verify the impact of the mutation on the splicing process. We used the genomic DNA of the proband or other normal family members as a template. Because the mutation is located after exon 1 of the SMARCAD1 gene and exon 1 does not encode, we directly used intron 1 and exon 2 in construction. In order to better simulate the real gene and ensure the constructed gene would not be misidentified, we added pseudoexon 1 and pseudoexon 2 in intron 1 (Figure 3).

The pseudoexon 1's sequence was ggagccaaaggtgaccgaggactgccagggccgcgaggcgagaag. The intron 1's sequence was gtgaggtgggttggccctggggcctgactactgagcagagaaggctcagtccagacacccctcacctgccattctgtgcag. The pseudoexon 2's sequence was ggtgaagctggccgtgcaggggagcccggagaccctggggaagat.

#### 2.5.2. PCR Amplification

PCR amplification reaction was performed by the PrimeSTAR® with GXL DNA Polymerase reagent instruction and digested with vector XhoI/EcoRI. We performed the recombination reaction according to the Hieff Clone™ Plus One Step Cloning Kit. We delivered the bacteria solution, which contains recombinant cloned products, to the Shanghai Genassistant Biotechnology Company Ltd. for sequencing. We obtained the wild-type plasmid pMini-SMARCAD1-WT and the mutant plasmid pMini-SMARCAD1-MUT by selecting monoclonal colonies and performing plasmid extraction.

RETRACTED

#### 2.5.3. Cell Transfection and Transcript Sequencing

Empty vector plasmids as well as wild-type and mutant type SMARCAD1 plasmids were transfected into 293 T cells. Cell observation was made under fluorescence microscope in 48 hours. After the transfection succeed, the cells were collected. Twice rinses were performed with precooled PBS. We added lytic cells and, after 30 minutes, performed RNA extraction and reverse transcription. PCR and electrophoresis were performed. We performed sequencing on the wild-type and mutant PCR products and analyzed differences in splicing.

## 3. Results

### 3.1. Pedigree Investigation

Among 28 family members (4 generations), there were total 12 individuals exhibiting a consistent skin phenotype (Figure 1). All affected individuals in this pedigree presented multiple milia on face at birth, which disappeared within 6 months. The recurrent blisters in extremities started at first month, which self-healed within a week and finally disappeared within a year. But after that, palmoplantar hyperkeratosis appeared and became more and more obvious along with the increasing in age (Figure 1(e)). With time, tapering of fingers and longitudinal ridges of nails gradually appeared (Figures 1(c) and 1(d)). No fingerprint could be seen in extremities and all the affected individuals exhibited no or less sweat in hands and feet. Hairs and teeth were normal. Consanguineous marriage was denied.

According to the family history inquiry, among the 5 individuals who have passed away in the 1st and 2nd generation, only 1 individual (II-5) died of brain stroke with obesity, hypertension, and gout at the age of 54, while the remaining 4 individuals died of multiple metastases of finger cSCC. II-7 was a tailor. He had several years' history of dorsal digital skin ulcer but never sought for any medical treatment. He finally visited the hospital due to the severe deterioration of the ulcer (finger bone exposing). He took a skin biopsy and was diagnosed as cSCC. He was hospitalized for a finger amputation in Zhuhai People's Hospital in 2010. Although underwent standard chemotherapy, 2 years later, he died of multiple metastasis including lung metastasis and spinal metastasis at 51 years old. II-3, born in 1959, was a blue-collar worker. He was admitted to Tongji Hospital for a nonhealing ulcer of the dorsal finger in 2012. A pathological diagnosis of cSCC was made after the skin biopsy. Axillary metastasis emerged soon after surgical resection of the tumor. Finally, he died of uncontrollable bleeding from axillary metastatic tumor at 57 years old. Two other family members (I-1 and II-1, an accountant and a blue-collar worker) had similar experience and died due to massive bleeding of axillary metastatic tumor at the ages 36 and 45, respectively.

RETRACTED

### 3.2. Mutation in the SMARCAD1 Gene

To identify the underlying pathological gene, we performed WES for the proband (IV-6). A heterozygous mutation in the SMARCAD1 gene NM_001254949.2: c.-10+5G>A (if counting from the beginning of the noncoding exon 1, this mutation would be named as c.378+5G>A) was identified. The WES result was further confirmed by Sanger sequencing (Figure 4(a)).

Sanger sequencing was also performed for III-2, III-6, III-10, III-11, IV-1, and IV-4. As shown in the pedigree chart (Figure 2), (+) indicates the mutation has been confirmed by Sanger sequencing. (-) indicates no mutation was detected by Sanger sequencing. III-2, III-6, III-10, and IV-4 were clinically diagnosed with Basan syndrome. They were also confirmed carrying the same mutation by Sanger sequencing.  Figure 4(b) illustrates the mutation of the proband's father (III-10). III-11 and IV-1 did not carry this mutation, while no Basan syndrome was diagnosed.  Figure 4(c) illustrates that the mutation was not discovered in the proband's mother (III-11). This revealed that the mutation cosegregated with Basan syndrome in this pedigree. Bioinformatics analysis showed that this mutation was not detected in the 1000 genome database, ExAC databases, or gnomAD database.

### 3.3. WES Results

#### 3.3.1. Quality of the WES Data

One of the 7 collected blood samples (III-2) was contaminated due to misoperation before performing WES. Therefore, WES was performed for only 6 individuals.  Table 1 summarizes the results. All of the 6 samples had a coverage higher than 98% at 4X. The average depth was 160.22 for III-6, 193.60 for III-10, 136.44 for III-11, 176.87 for IV-1, 157.72 for IV-4, and 136.29 for IV-6. In summary, the sequencing data had reached the required quality for next step analysis.

#### 3.3.2. SMARCAD1 and Other Gene Mutation Analyses in WES

Based on the WES data, we performed target analysis for the SMARCAD1 gene to further confirm the association between SMARCAD1 and Basan syndrome. As shown in Table 2, all Basan syndrome patients carried the mutation SMARCAD1, chr4: 94253676G>A. Specifically, III-6 had 63 reads mapped to SMARCAD1 variant with a frequency of 0.406; III-10 had 60 reads mapped with a frequency of 0.400; IV-4 had 66 reads mapped with a frequency of 0.485; and IV-6 had 54 reads mapped with a frequency of 0.519. Other family member who was not diagnosed with Basan syndrome did not carry this mutation.

RETRACTED

As described above, the family history revealed 4 affected members with cSCC in the 1st and 2nd generations. This family exhibited high cooccurrence rate between Basan syndrome and cSCC. To discover the potential highly related gene mutations, we further investigated WES results in the ClinVar database and COSMIC database, aiming for cancer-related gene mutations. Due to the limited samples available, we set out to apply strict filtering criteria for finding possible associated gene mutations. The criteria only kept mutations occurring in the four individuals with Basan syndrome (III-6, III-10, IV-4, and IV-6) but not in other two non-Basan individuals (III-11 and IV-1). The results from the filtering criteria retained 3434 mutations. Out of these 3434 mutations, only one mutation, rs751141, was mapped to the ClinVar database. The annotation of rs751141 shows that it is a risk factor related to “hypercholesterolemia, familial.”

The above-mentioned 3434 mutations were then mapped in the COSMIC database. In order to find more significance related to the FAMILIAL cancer, we only retained the exonic area and presented as “nonsynonymous” or “frameshift.” After filtering, three genetic variants appeared in individuals with Basan syndrome but not in non-Basan individuals: rs3085861 (SETBP1), rs663651 (SETBP1), and rs2454206 (TET2). Both SETBP1 gene and TET2 gene have been reported associating with skin cancers, including cSCC [14]. However, according to dbSNP, all of the three genetic variants observed in this study are common variants.

#### 3.3.3. Functional Analysis

Minigene was preformed to further analyze the SMARCAD1 pre-mRNA splicing. We constructed a Minigene containing genomic sequence from intron 1, pseudoexon 1, pseudoexon 2, and exon 2. Our data indicated that the mutation in the SMARCAD1 gene site can lead to splicing variations: pseudoexon 1, pseudoexon 2, and exon 2 were all detected in the wild type, but pseudoexon 2 was skipped in the mutation type (Figure 5). This mutation was located in the intron 1. No other potential splicing site was found. The Minigene result demonstrated that this mutation in intron 1 may cause the gene-splicing variation. Contrarily, no mutation in the intron (wild-type) exhibited normal expression of pseudoexon 1, pseudoexon 2, or exon 2.

## 4. Discussion

In this study, we reported a new Chinese pedigree with Basan syndrome and family history of cSCC. We identified the pathogenic mutation site in the SMARCAD1 gene. To the best of our knowledge, this is the 15th Basan syndrome case reported in the world, and the first reported Basan syndrome pedigree with history of cSCC.

RETRACTED

The mode of inheritance in the pedigree reported here is autosomal-dominant inheritance. Its clinical symptoms are in line with the typical clinical manifestations of Basan syndrome, which belongs to the supporting evidence (PP4). Its mutation site is c.378+5G>A in SMARCAD1, which is identical to the case of Basan syndrome reported in Chang [7]. This mutation site has not been reported in the public databases of human mutation, such as ExAC, 1000G, and gnomAD. It is a rare mutation and belongs to the moderate pathogenicity evidence (PM2). This mutation was detected in multiple patients in the family, which belongs to the supporting evidence (PP1-Moderate). With the verification by Minigene, we found that it may cause splicing variation, which belongs to the strong pathogenicity evidence (PS3-Moderate). According to the Genetic Variant Classification published by the American College of Medical Genetics and Genomics (ACMG), this mutation type should be classified as a potential pathogenicity to Basan syndrome.

SMARCAD1 is a member of the chromatin remodeling ATPase of SNF2 helicase superfamily, located at 4q22 [2]. It is widely expressed in 27 normal human tissues, including thyroid, testis, and skin [15]. It has been discovered that the SMARCAD1 gene has two isoforms with different transcription starting sites. The long isoform contains 24 exons expressed. It encodes 1028 amino acid proteins. It is widely expressed at a low level. The short isoform, as known as the skin-specific isoform, is mostly expressed on skin fibroblasts and keratinocytes [7]. SMARCAD1 is a transcription factor. It participates in many biological processes. It may be involved in dermatoglyph and sweat gland development by regulating the expression of epidermal differentiation-associated genes [16]. In addition, it also plays an import role in repairing potentially lethal DNA double-strand breaks [13] and maintaining genome integrity by stabilizing active replication [17]. Multiple studies have demonstrated that break points and mutations of the gene are involved in several human diseases, such as genodermatosis [5, 18, 19], malignant peripheral nerve sheath tumors [20], breast cancer [17], and pancreatic cancer [21].

Besides Basan syndrome, there are two other phenotypes of genodermatosis related to the SMARCAD1 gene: adermatoglyphia and Huriez syndrome. Adermatoglyphia (OMIM: 136000) is clinically characterized by no fingerprint, mildly clubbed finger, and less or no sweat on the palmoplantar due to decreased number of sweat glands [22]. Mutations (c.378+1G>T, c.378+2T>C, c.378+5G>C, and c.378+1G>A) in the SMARCAD1 gene were found to be associated with this disease [16, 18]. Huriez syndrome (OMIM: 181600) is another rare autosomal-dominant genodermatosis, which shows three serial clinical manifestations: congenital sclerosis and atrophy at the end of extremities, palmoplantar keratoderma, and nail dysplasia. One feature of this disease is the risk of 15% to develop aggressive cSCC in the affected skin region at age 30 to 50 [23]. The cSCC in Huriez syndrome seems to be more aggressive and more likely to develop metastases than usual cSCC [24]. Huriez syndrome was first recognized in 1963 by Huriez and coworkers. But the causative SMARCAD1 gene was only characterized for a few years due to the rarity of the disease [25]. Till now, related mutation sites, including c.378+2T>C, c.378+2_3insT, c.363_378+2del, and NC_000004.12:g.94252297_94253585del, were screened in the SMARCAD1 gene [19, 25].

RETRACTED

From the perspective of clinical characteristics (listed in Table 3), adermatoglyphia, Basan syndrome, and Huriez syndrome have similarities: mild palmoplantar keratoderma, less or no sweat in the palmoplantar region, and finger flexion contracture. However, clinical manifestations of adermatoglyphia do not include blister or milia. Patients with adermatoglyphia have normal nails. For Basan syndrome, patients are vulnerable to milia and blisters. Patients with Huriez syndrome are more vulnerable to cSCC, skin heterochromia, hand sclerosis and atrophy, and thin fingers. As shown in Table 3, adermatoglyphia and Basan syndrome share the same mutation site in the SMARCAD1 gene: c.378+1G>T. Adermatoglyphia and Huriez syndrome share the same mutation site: c.378+2T>C. We suspect that adermatoglyphia, Basan syndrome, and Huriez syndrome belong to the same disease spectrum, while adermatoglyphia is the mildest and Huriez syndrome is the most severe. Some researchers hypothesize that the risk of cSCC would increase if a patient presents both adermatoglyphia and Basan syndrome [25]. However, there is no such reported case due to the rarity of these diseases.

Four of twelve members in the reported pedigree with Basan syndrome died due to hand cSCC metastasis. This demonstrates the potential association between cSCC and Basan syndrome, which is partially in line with Gunther's hypothesis [25]. In this study, we investigated gene mutations through WES aiming to verify the potential association between cSCC and Basan syndrome. We located three genetic variants shared by individuals with Basan syndrome but not by non-Basan individuals in the pedigree. The corresponding mutant genes have been reported associating with skin cancers, including cSCC [14]. However, these three genetic variants are common variants reported in dbSNP. Therefore, we currently cannot draw any conclusion about the association between cSCC and Basan syndrome. There are several reasons account for this issue. Foremost, even we succeeded in examining most available Basan patients in this pedigree, the number of cases is still small. In addition, due to the 4 cSCC patients had passed away for years, we failed to acquire their tissues from the local hospitals. These are main limitations in this study. Nevertheless, with the high incidence rate of cSCC in this Basan syndrome pedigree, we believe that this potential association is worth to be evaluated in future studies, especially roles and mechanisms of SMARCAD1 gene mutations in tumorigenesis and metastasis.

RETRACTED

In conclusion, we discovered a new Chinese pedigree with Basan syndrome and family history of cSCC. We confirmed a gene mutation in the SMARCAD1 gene c.378+5G>A and expanded the disease spectrum. Minigene results showed the mutation at the intron may cause splicing variations. We also intended to assess the potential association between Basan syndrome and cSCC. Despite currently we cannot draw any conclusion, this report encourages future works to substantiate this potential but important issue.

## Figures and Tables

**Figure 1:** Clinical presentation of the proband and her father: (a) multiple eruptive milia appeared on the chin when the proband was born; (b) hyperkeratosis, skin atrophy, and mild pigmentation in the palmar region of the proband; (c) tapering of fingers and no fingerprint in the extremity of the proband's father; (d) longitudinal ridges of nails of the proband's father; and (e) obvious hyperkeratosis in the plantar region of the proband's father.

**Figure 2:** Pedigree chart. Individuals highlighted in black had Basan syndrome. (+) indicates the mutation in the SMARCAD1 gene had been confirmed by Sanger sequencing. (-) indicates no mutation in the SMARCAD1 gene was detected by Sanger sequencing.

**Figure 3:** An illustration of plasmid construction. Pseudoexon 1 and pseudoexon 2 were introduced exogenously to construct the Minigene.

**Figure 4:** Sanger sequencing result of the pathogenic mutant gene of the (a) proband, (b) proband's father, and (c) proband's mother.

**Figure 5:** An illustration of Minigene analysis.

**Table 1:** Whole exome sequencing results.

	III-6	III-10	III-11	IV-1	IV-4	IV-6
Raw data base (GB)	14.98	18.48	13.13	16.31	14.76	12.88
Raw data reads	149,843,780	184,800,454	131,389,028	163,159,766	147,678,418	128,884,472
Clean data base (GB)	14.77	18.21	12.9	16.13	14.55	12.65
Clean data reads	148,997,060	183700867	130,066,438	162,540,046	146,819,461	127,529,011
Target reads	100,052,692	123,297,215	84,700,803	109,486,188	99062265	83,651,114
Fraction of target reads in mapped results	67.15%	67.12%	65.12%	67.36%	67.48%	65.59%
Average depth	160.22	193.60	136.44	176.87	157.72	136.29
Coverage (≥4x)	98.42%	98.43%	98.27%	98.24%	98.42%	98.24%
Coverage (≥10x)	98.29%	98.28%	98.09%	98.08%	98.23%	98.06%
Coverage (≥30x)	97.40%	97.23%	96.62%	96.95%	96.74%	96.45%
Coverage (≥100x)	80.17%	82.85%	70.65%	80.84%	77.43%	69.84%

RETRACTED

**Table 2:** SMARCAD1 mapped reads.

	III-6	III-10	III-11	IV-1	IV-4	IV-6
SMARCAD1						
Ref-depth	92	90	132	135	70	50
Alt-depth	63	60	0	0	66	54
AF	0.406	0.400	0	0	0.485	0.519

**Table 3:** Summary of phenotypes and mutation types related to mutations in the SMARCAD1 gene.

Reference	Adermatoglyphia	Basan syndrome					Huriez syndrome
	2011 Burger [22]	2014 Mark [5]	2018 Valentin [2]	2016 Li [6]	2018 Chang [7]	Pedigree reported in this study	2021 Loh [19]
Milia on the chin	—	+	+	+	++	+	—
Nonfingerprint	+	+	+	+	++	+	+
Finger flexion contracture	+	—	—	+	++	Mild	+
Blisters or erosions	—	+	+	+	++	+	—
Hyperkeratosis at the pressured palmoplantar area	+	—	+	2/8	—	+	+
Nail disease	—	—	—	Onychodystrophy 1/8	—	Longitudinal ridges	Longitudinal ridge and hypoplasia, thin fingers
Palmoplantar pigmentation spots	—	—	+	5/8	—	Mild	—
Less or no sweat	+	++	—	+	—	+	+
Other clinical manifestations	—	—	—	Knuckle pads 7/8	Bilateral syndactyly	Tapering of the fingers	Scleroatrophy of the hands, tapering of the fingers, and poikiloderma of the nose
Autosomal-dominant inheritance	+	+	No family history	+	++	+	+
Mutation types in the SMARCAD1 gene	c.378+1G>T [18] c.378+1G>A c.378+2T>C c.378+5G>C [16]	c.378+3A>T	c.378+2T>G	c.378+1G>T	45-kb heterozygous deletion (chr4:95,129,542-95,174,582), c.378+5G>A	c.378+5G>A	NC_000004.12:g.94252297_94253585del [19] c.378+2T>C, c.378+2_3insT [25], c.363_378+2 del [25]

## Data Availability

The data used in this research are available from the corresponding author upon reasonable request.

## References

[1] Baird H. W. (1964). Kindred showing congenital absence of the dermal ridges (fingerprints) and associated anomalies. *The Journal of Pediatrics*.

[2] Valentin M. N., Solomon B. D., Richard G., Ferreira C. R., Kirkorian A. Y. (2018). Basan gets a new fingerprint: mutations in the skin-specific isoform of SMARCAD1 cause ectodermal dysplasia syndromes with adermatoglyphia. *American Journal of Medical Genetics. Part A*.

[3] Basan M. (1965). Ektodermale Dysplasie. *Archiv für Klinische und Experimentelle Dermatologie*.

[4] Reed T., Schreiner R. L. (1983). Absence of dermal ridge patterns: genetic heterogeneity. *American Journal of Medical Genetics*.

RETRACTED

[5] Marks K. C., Banks W. R., Cunningham D., Witman P. M., Herman G. E. (2014). Analysis of two candidate genes for Basan syndrome. *American Journal of Medical Genetics. Part A*.

[6] Li M., Wang J., Li Z. (2016). Genome-wide linkage analysis and whole-genome sequencing identify a recurrent SMARCAD1 variant in a unique Chinese family with Basan syndrome. *European Journal of Human Genetics*.

[7] Chang X., Li D., Tian L. (2018). Heterozygous deletion impacting SMARCAD1 in the original kindred with absent dermatoglyphs and associated features (Baird, 1964). *The Journal of Pediatrics*.

[8] Limova M., Blacker K. L., LeBoit P. E. (1993). Congenital absence of dermatoglyphs. *Journal of the American Academy of Dermatology*.

[9] Cirillo-Hyland V. A., Zackai E. H., Honig P. J., Grace K. R., Schnur R. E. (1995). Reevaluation of a kindred with congenital absence of dermal ridges, syndactyly, and facial milia. *Journal of the American Academy of Dermatology*.

[10] Nieto-Benito L. M., Molina-Lopez I., Feito-Rodriguez M., Martinez-Gonzalez V., Suarez-Fernandez R., Campos-Dominguez M. (2021). Ectodermal dysplasia with congenital adermatoglyphia (Basan syndrome): report of two cases presenting with extensive congenital milia. *Pediatric Dermatology*.

[11] Luna P. C., Larralde M. (2012). Profuse congenital familial milia with absent dermatoglyphics (Basan's Syndrome): description of a new family. *Pediatric Dermatology*.

[12] Jorgenson R. (1974). Ectodermal dysplasia with hypotrichosis, hypohidrosis, defective teeth, and unusual dermatoglyphics (Basan syndrome?). *Birth Defects*.

[13] Costelloe T., Louge R., Tomimatsu N. (2012). The yeast Fun30 and human SMARCAD1 chromatin remodellers promote DNA end resection. *Nature*.

[14] AACR Project Genie Consortium (2017). AACR project GENIE: powering precision medicine through an international consortium. *Cancer Discovery*.

[15] Fagerberg L., Hallström B. M., Oksvold P. (2014). Analysis of the human tissue-specific expression by genome-wide integration of transcriptomics and antibody-based proteomics. *Molecular & cellular proteomics: MCP*.

[16] Nousbeck J., Sarig O., Magal L. (2014). Mutations in SMARCAD1 cause autosomal dominant adermatoglyphia and perturb the expression of epidermal differentiation-associated genes. *The British Journal of Dermatology*.

[17] Lo C. S. Y., Mv T., Gaggioli V. (2021). SMARCAD1-mediated active replication fork stability maintains genome integrity. *Science Advances*.

[18] Nousbeck J., Burger B., Fuchs-Telem D. (2011). A mutation in a skin-specific isoform of SMARCAD1 causes autosomal-dominant adermatoglyphia. *American Journal of Human Genetics*.

[19] Loh A., Ho C., Muthiah S. (2021). Huriez syndrome caused by a large deletion that abrogates the skin-specific isoform of SMARCAD1. *British Journal of Dermatology*.

RETRACTED

[20] Han H., Jiang G., Kumari R. (2021). Loss of smarcad1a accelerates tumorigenesis of malignant peripheral nerve sheath tumors in zebrafish. *Genes, Chromosomes & Cancer*.

[21] Liu F., Xia Z., Zhang M. (2019). SMARCAD1 promotes pancreatic cancer cell growth and metastasis through Wnt/*β*-catenin-mediated EMT. *International Journal of Biological Sciences*.

[22] Burger B., Fuchs D., Sprecher E., Itin P. (2011). The immigration delay disease: adermatoglyphia-inherited absence of epidermal ridges. *Journal of the American Academy of Dermatology*.

[23] Lee Y. A., Stevens H. P., Delaporte E., Wahn U., Reis A. (2000). A gene for an autosomal dominant scleroatrophic syndrome predisposing to skin cancer (Huriez syndrome) maps to chromosome 4q23. *American Journal of Human Genetics*.

[24] Guerriero C., Albanesi C., Girolomoni G. (2000). Huriez syndrome: case report with a detailed analysis of skin dendritic cells. *The British journal of dermatology*.

[25] Gunther C., Lee-Kirsch M. A., Eckhard J. (2018). SMARCAD1 haploinsufficiency underlies Huriez syndrome and associated skin cancer susceptibility. *The Journal of Investigative Dermatology*.

